# Artificial Intelligence Segmentation Algorithm-Based Optical Coherence Tomography Image in Evaluation of Binocular Retinopathy

**DOI:** 10.1155/2022/3235504

**Published:** 2022-06-01

**Authors:** Jiemei Shen

**Affiliations:** Department of Ophthalmology, The First People's Hospital of Tonglu County, Tonglu, 311500 Hangzhou, China

## Abstract

On account of optical coherence tomography (OCT) images with intelligent segmentation algorithm, this article investigated the clinical efficacy and safety of docetaxel combined with fluorouracil. In this study, 60 patients with retinopathy treated in hospital were selected as the research objects. There were 30 cases in each group, the control group was treated with conventional images, and the observation group was treated with algorithm-based OCT images. Intelligent segmentation boundary detection algorithm, boundary tracking, and contour localization were proposed and applied to the OCT images of patients to analyze features and measure corneal thickness in OCT images with high signal-to-noise ratio and noise and artifacts. Objects in the control group were treated with semiconductor laser, and those in the observation group were treated with OCT images with algorithm in addition to the treatment of the control group. The results showed that the number of images with relative error of 2 was more, and the number of images with relative error of -2 was the least. The average thickness of high-quality images was 562.7 *μ*m, and the average thickness of images with noise and artifacts was 573.8 *μ*m. The total effective rate of the observation group was 96.67%, which was significantly higher than that of the control group (80%), and the curative effect and physical improvement rate of the observation group were significantly better than that of the control group (*P* < 0.05). All in all, the feature extraction of OCT images and corneal measurement proposed in this study had a good measurement effect, and the method had the advantages of strong anti-interference ability and high measurement accuracy.

## 1. Introduction

The retina is also the fundus. There are very important visual tissues on the retina, such as macula and optic nerve. Once the retinal lesions occur in both eyes, the vision of patients will be very poor, such as optic nerve atrophy, macular degeneration, optic neuritis, and retinitis pigmentosa [1, 2]. Clinically, there is a wide range of retinopathy, many of which are treated with specific drugs. However, binocular retinopathy is a genetic disease which is difficult to use effective drugs to treat [3, 4]. The factors causing retinopathy are relatively complex, and different cases are analyzed according to the specific situation [5, 6].

Optical coherence tomography (OCT) is a new tomography technology with the most promising and rapid development in recent years, especially in biological tissue in vivo detection and imaging, which has attractive application prospects [7]. It has been tried to be applied in clinical diagnosis of ophthalmology, dentistry, and dermatology [8, 9]. OCT is a new optical diagnostic technique that enables noncontact and noninvasive tomography of living tissue microstructure [10, 11]. In a highly sensitive detection technique, OCT enables the acquisition of clear tomographic images in light scattering media with a resolution of 1-15 *μ*m. OCT is an optical simulation of ultrasound. Its axial resolution depends on the coherence characteristics of the light source, up to 10 meters, and the penetration depth is almost not limited by inflammatory transparent refractive media. It can observe the anterior segment and display the morphological structure of the posterior segment of the eye [12, 13].

OCT imaging devices can quickly and contiguously obtain high-resolution sectional images of the anterior segment and accurately measure the thickness of the central cornea [14, 15]. However, in OCT imaging equipment, the light source, detection circuit, galvanometer, and multiple scattering of light in practical application will cause serious noise, resulting in the appearance of weak corneal edge, which seriously affects the extraction of central corneal contour and thickness calculation. Sinclair et al. (2015) [16] used pixel-level edge detection to extract the internal and external corneal contour, but the obtained corneal contour was not smooth enough and was susceptible to noise and weak edge, with certain defects in stability. Coron et al. (2007) [17] extended the extraction algorithm for the contour of the anterior chamber of the eye in ultrasound images to OCT images. The iterative method was used to remove the interference of the central bright line.

In order to supply a gap in PCT imaging, an automatic measurement algorithm of central corneal thickness on account of edge detection and random sample consensus (Ransac) was proposed in this study to reduce the noise in the image, remove the OCT artifacts of the cornea, and strengthen low SNR regional robust. The upper and lower boundaries of the central cornea were detected by the boundary detection operator. The upper and lower boundaries of the central cornea were obtained by Ransac arc fitting algorithm. The thickness of the central cornea was determined, so as to provide reference for clinical diagnosis of retinopathy.

## 2. Materials and Methods

### 2.1. Study Subjects

In this study, 60 patients with retinopathy who were admitted to hospital from May 2019 to December 2020 were retrospectively analyzed. The patients were randomly divided into two groups according to their own will. The control group (*n* = 30) included 12 male patients and 18 female patients, aged from 33 to 65 years old, with an average age of 51.0 ± 3.2 years old. In the observation group (*n* = 30), there were 13 males and 17 females, aged from 34 to 61 years old, with an average age of 57.8 ± 3.4 years old. The general data of the two groups were comparable, and there was no statistical significance (*P* > 0.05). This study was approved by ethics committee of hospital, and patients and their families were informed of the study and signed informed consent.

Inclusion criteria: first, the patients were diagnosed with retinopathy after examination. Second, the patients agreed to join the study. Third, the patients were from 30 to 70 years old. Fourth, the patients could communicate normally, without linguistic barriers.

Exclusion criteria: first, patients contraindicated with OCT scanning. Second, patients with vascular dementia, lewy body dementia, and other mental diseases. Patients with incomplete clinical data and imaging data. Fourth, women in lactation or pregnancy.

### 2.2. Treatment Methods

In the control group, the semiconductor laser pumped frequency doubling laser was used. The spot diameter was 200-300 *μ*m, the wavelength was 532 nm, and the exposure time was 0.1-0.2 s. Local photocoagulation was performed for localized macular edema, and diffuse edema was more than 500 *μ*m away from the fovea. Patients with proliferative retinopathy were treated with an extensive retinal beam four times a week. On the basis of the treatment of the control group, the observation group was treated with OCT images introduced with algorithm. During OCT detection, the lower jaw was placed on the bracket in the sitting position, and the central point of the optic disc was selected with a diameter of 3.45 mm. A 360° circular scan was performed. Computer image intelligence analysis tools automatically measure retinal thickness. Mean retinal thickness, central thickness, and retinal relative error were recorded. The denoising and edge denoising results of the OCT image were observed, and the image edge fitting effect was analyzed. Finally, the treatment effect of the two groups of patients was analyzed.

### 2.3. Central Corneal Thickness Automatic Measurement Algorithm on Account of Ransac and Edge Detection

The image quality is uneven. Some images show low contrast, blurred boundaries, and small targets. The size and shape are changeable. The pixels are close to blood vessels and other tissues in the tissue. It is easy to distinguish highly similar features in the image, which also increases the difficulty of image segmentation. The OCT imaging quality of the anterior segment varies according to the objective environment and imaging objects. Many images exist serious noise, causing the appearance of weak boundaries, while some images are interfered by the central bright line, and the upper and lower edges of the cornea are not smooth enough. The process diagram of the automatic measurement algorithm of central cornea thickness on account of Ransac and edge detection was shown in Figure 1. First, the image is preprocessed, and the central corneal upper edge is fitted by the Ransac algorithm, then, the corneal edge is extracted, and finally, the central corneal thickness is calculated.

### 2.4. Basic Algorithm

The automatic measurement method of corneal thickness can not only measure corneal thickness of high-quality corneal images but also accurately measure OCT images with more noise and artifacts in the images. The general flow chart of this measurement method was shown in Figure 2. First, OCT images were preprocessed using adaptive median filtering and artifacts, binarization was used to process the images, and boundary tracking algorithm was used to obtain the upper and lower edge contour points. Second, the upper and lower edges of the cornea could be fitted by the least square method according to the upper and lower edges of the cornea, the cornea coordinates of the whole image could be obtained. Third, the cornea thickness could be calculated by the coordinate points. Finally, the accurate data could be obtained.

### 2.5. Adaptive Median Filtering

Image preprocessing is to eliminate the interference of noise and different artifacts on automatic measurement of corneal thickness. Adaptive median filtering and artifact removal can avoid image edge blur. When the probability of noise occurrence is less than 0.2, the median filter can remove the noise well. When the probability is larger, the noise is more obvious. As illustrated in Figure 3, adaptive median filtering was able to deal with impulsive noise with a greater probability and retain details as much as possible while balancing nonimpulsive noise. Adaptive median filtering included whether the median point of the current window was noisy and whether the pixel at the center of the window was noisy. When judging whether there was noise at the median point, it was suggested to increase the window size of the filter and looked for a nonnoise median in a larger range. In order to return to find the median, the size of the window should reach the maximum value.

### 2.6. Boundary Tracking Algorithm

The boundary tracking algorithm refers to the boundary between a pixel connected domain and 0 pixel connected domain and extracts a series of coordinate points of the boundary contour. Pixels with grayscale values of 0 and 1 are called 0 pixel and 1 pixel. If 0 pixel fills the border of the binary image, any value can be given to the pixel in the processing. The four boundaries of a binary image form the border of an image. Pixel points in row *X* and column *Y* were represented by (*X*, *Y*), and gray value *G*_*xy*_ of image pixel points at (*X*, *Y*) was defined as

(1) $$\begin{array}{c} G=\left(G_{xy}\right). \end{array}$$

If the binary image is scanned line by line until the condition (*X*, *Y*) meets the starting point of boundary tracking is found, the scanning is stopped. The schematic diagram of outer boundary and inner boundary was shown in Figure 4.

If the input image is *W*, the frame of *W* forms a special empty hole boundary, and the matching sequence is set to 1, then *W*_*NB*_ = 1, and *W*_*NB*_ represents the current boundary sequence number. If (*X*_3_, *Y*_3_) represents the current point, and (*X*_2_, *Y*_2_) represents the point preceding the current point, each time a new row is scanned again.

For the steps satisfying the scan graph, the first step is to determine that the pixel is an outer boundary tracking starting point, and the *W*_*NB*_ increases with (*X*, *Y*_−1_)⟶(*X*_2_, *Y*_2_). In the case of *Gxy* ≥ 1 and *Gx*, *y* − 1 = 0, then, it is determined that pixel (*X*, *Y*) is the starting point of a hole boundary and *W*_*NB*_ increases with (*X*, *Y*_+1_)⟶(*X*_2_, *Y*_2_). The border type and the border type with the serial number determine the parent border of the front border.

1. It is suggested to start with (*X*_2_, *Y*_2_) and search the neighborhood of (*X*, *Y*) clockwise to find a nonzero. (*X*_1_, *Y*_1_) is the first nonzero, if no nonzero is found, step jump will be performed
2. (*X*, *Y*)⟶(*X*_3_, *Y*_3_) and (*X*_1_, *Y*_1_)⟶(*X*_2_, *Y*_2_)
3. In the neighborhood of the current point (*X*_3_, *Y*_3_), the next element from the counterclockwise starting point is (*X*_2_, *Y*_2_), and the next element to look for can be set to (*X*_4_, *Y*_4_)
4. It is suggested to change the value of points (*X*_3_, *Y*_3_), *GX*_3_, *Y*_3_, according to the rule
5. (*X*_4_, *Y*_4_) = (*X*, *Y*) and (*X*_3_, *Y*_3_) = (*X*_1_, *Y*_1_) go to the previous step, otherwise, (*X*_4_, *Y*_4_) (*X*_3_, *Y*_3_) and (*X*_4_, *Y*_4_) (*X*_2_, *Y*_2_) and go back to step 3

If *Yxy* is not equal to 1, there will be a ∣*Gx*_*y*_ | ⟶*Wl*_*NB*_ rescanning point is (*X*, *Y* + 1), when the scanning to the lower right corner, algorithm runs over.

### 2.7. Automatic Measurement of Corneal Thickness

Some noises and unerased artifacts in Figure 5 seriously affected the extraction of corneal contour points. After the contour of the image was obtained by using the boundary tracking method, the minimum tangent rectangle of the cornea was found, the upper and lower boundaries of the cornea were fitted by using the most child method.

If the fitting curve equation of the upper corneal boundary is

(2) $$\begin{array}{c} Y1=a1x_{1}^{2}+b_{1}x_{1}+C_{1}, \end{array}$$

(3) $$\begin{array}{c} Y_{2}=a_{2}x_{2}^{2}+b_{2}x_{2}+C_{2}. \end{array}$$

Any point was chosen as *E*_1_ (*x*_1_, *y*_1_), and the corresponding point on the corneal margin was *E*_2_ (*X*_2_, *y*_2_), which was the same as the abscissa of the change point. OCT images were obtained by fourier transform of the real part of the interference spectrum, forming a tomographic image including the sample itself, and a symmetric mirror image with zero phase delay. Within the depth range of system imaging, half of the sampling points are used for each A-scan. Each A-scan sampling point is represented by *N*, and the system imaging depth is represented by *h*.

Equation *H* of corneal thickness is

(4) $$\begin{array}{c} D=\frac{2\left(y_{2}-y_{1}\right)h}{N}. \end{array}$$

### 2.8. Experimental Environment

In this study, the optical coherence tomography system was used to obtain OCT data of human cornea. The signal-to-noise ratio (SNR) of the system was 51 dB, the sensitivity was 101 dB, the central wavelength of the system light source was 1060 nm, the imaging depth was 3.7 mm, the longitudinal resolution was 7.5 *μ*m, and the lateral resolution was 57.0 *μ*m. For each OCT corneal image B-scan, there were 360 A-scans, and the sample number of A-scans was 1820. The size of B-scan images of OCT images selected was 360 pixel × 360 pixel. As experimental data, high-quality OCT images of cornea were selected in a 3.4 GHz central processing unit (CUP), and the corneal thickness was automatically measured by random access memory on a 4.0 GB computer.

### 2.9. Statistical Methods

SPSS19.0 statistical software was used to analyze the survey data in this study. Mean ± standard deviation (^−^*x* ± *s*) was used to represent the measurement data conforming to normal distribution, and frequency and frequency (%) were used to represent the nonconformity count data. *T*-test data and chi-square test were used for quality comparison. *P* < 0.05 was statistically significant, and vice versa.

## 3. Results

### 3.1. OCT Images

As shown in Figure 6, OCT image was from a man, 43 years old. Figure 6 showed that there was noise in the original image in Figure 6(a), because the imaging process was disturbed by light sources, circuits, light scattering, etc. The denoised image in Figure 6(b) was obtained by using the median filter in the algorithm. The boundary detection operator was used to extract the existing edges in the image, and the edge extracted image was obtained. As could be understood from the image, if feature extraction was carried out directly, the image effect was not ideal.

### 3.2. Image Fitting Results

In Figure 7, OCT image was from a woman, 51 years old. Figure 7(a) is the OCT image with noise and artifacts, and Figure 7(b) is the edge fitting image of B-scan corneal image with noise and artifacts.

### 3.3. Corneal OCT Image Thickness Comparison

Curve fitting results of high-quality OCT images and OCT images with noise and artifacts showed that the average thickness of the high-quality image was 562.7 *μ*m, and the average thickness of the image with noise and artifacts was 573.8 *μ*m. The average thickness of the high-quality image 8 was 573.8 *μ*m, and the average thickness of the image with noise and artifacts was 574.8 *μ*m. The average thickness and central thickness of the images with noise and artifacts were higher than those of OCT scans with better image quality, as given in Figure 8.

### 3.4. Relative Error of Retina

Different numbers of images were selected to compare relative errors. As shown in Figure 9 that the number of pictures with relative error of 2 was relatively large, followed by that with relative error of 0 and that with relative error of -2 was the least.

### 3.5. Effect Comparison

The efficacy of the two groups was compared. As shown in Figure 10, the total effective rate of the observation group was 96.67%, significantly higher than that of the control group (80%), and the difference was statistically significant (*P* < 0.05, *χ*^2^ = 5.103).

## 4. Discussions

The pathogenesis of retinopathy is quite complex, and the main pathologies include thickening of the basal layer, proliferation of endothelial cells, and selective loss of pericytes. At present, the pathogenesis of retinopathy has not been clearly clarified. The photocoagulation effect of laser destroys part of the outer omentum with strong metabolism, thus, reducing the oxygen consumption of the retina [18]. Laser can make the retina thin, and then conducive to oxygen from choroid circulation to the inner layer of the retina, further mountain retinal microcirculation, the formation of neovascularization pair is reduced, avoid the retina. OCT is a very intuitive detection method and a good new imaging technology, which can observe three-dimensional cross-sectional images quantitatively and qualitatively and reflect the diagnosis and treatment of macular disease in detail [19]. Tzaridis et al. (2019) [20] showed in his study of retinopathy that binocular suppression of reading might be caused by a central dark spot unique to a noncorresponding retinal region. Medical imaging segmentation is to use digital instruments for quantitative and qualitative analysis of the pathological tissues in the image and to achieve three-dimensional model reproduction of the special tissues or objects in the image. How to segment medical image data accurately and quickly and optimize the segmentation effect is the key to image segmentation at the present stage [21]. Threshold segmentation method is to use one or more thresholds to divide the gray level of the image into several parts. Threshold segmentation can achieve effective image segmentation due to the large differences between the gray value or characteristic value of the image, but it is suitable for image segmentation with strong target and background pairs [22, 23]. Boundary detection is to divide the boundary into different regions according to the discontinuity or abruptness of the local feature values of adjacent pixels in the image. Boundary detection has no obvious medical image segmentation effect on target and background. There are mean filtering, median filtering, and Gaussian filtering in image denoising methods. Although Gaussian filtering can suppress the noise that follows normal distribution, it cannot remove speckle well. Median filtering is easy to lead to image discontinuity, and the effect of mean filtering to reduce noise is limited [24, 25]. Courrier et al. (2021) [26] used an efficient image analysis algorithm to analyze dry eye syndrome and stained the conjunctiva. The red channel was extracted from the original image, and the stained area was detected by the Gassapra filter. The threshold was manually determined on the image subset, and parameters in the algorithm remained unchanged. This algorithmic approach to image analysis and subjective evaluation suppression could provide clinical automation and scalability advantages. Elsawy et al. (2020) [27] used a new algorithm to flatten OCT images using air-epithelia. The mean value and segmentation time of operator errors were 0.89 ± 1.03 and 0.77 ± 0.68, respectively. The algorithm could generate accurate segmentation and thickness measurement. In this study, the average thickness of OCT images was 562.7 *μ*m using automatic corneal measurement, while that of images with noise and artifacts was 573.8 *μ*m. The central thickness of both images was higher than the average thickness, while that of images with noise and artifacts was higher than that of images with noise and artifacts. After the algorithm proposed in this study, the total effective rate of patients was 96.67%, which reflected that the algorithm proposed in this study could have a high segmentation and thickness measurement.

## 5. Conclusions

In this study, an automatic measurement method of central corneal thickness on account of the consistency of edge detection and random sampling was proposed. The initial edge in the OCT image of ocular segment histology was fitted by edge detection operator, and the upper edge of central cornea was fitted by algorithm to obtain the corneal thickness of the upper edge of central cornea. The total effective rate of patients using the algorithm in OCT images was 96.67%, significantly higher than that of the control group. The intelligent segmentation algorithm proposed in this study had good recognition efficiency for feature information segmentation of OCT images. The algorithm could effectively eliminate the noise in the image and accurately extract the central corneal edge. The limitation of this study is that the sample size is small, and the segmentation of image feature information cannot reach 100%. The follow-up work needs to expand the sample size to ensure the extensive application of the system. In conclusion, the algorithm model of this study can provide a theoretical basis for the extraction of ocular lesions features from OCT images in the medical system.

## Figures and Tables

**Figure 1:** OCT system imaging flowchart.

**Figure 2:** Flow chart of corneal measurement method.

**Figure 3:** Schematic diagram of adaptive median filtering process.

**Figure 4:** Boundary conditions. (a) Outer boundary. (b) Inner boundary.

**Figure 5:** Schematic diagram of automatic corneal thickness measurement.

**Figure 6:** OCT images.

**Figure 7:** Schematic diagram of corneal B-scan OCT image fitting.

**Figure 8:** Comparison of thickness of OCT images of different qualities.

**Figure 9:** Retinal relative error.

**Figure 10:** Comparison of curative effects between observation group and control group. ∗ suggested significant difference, *P* < 0.05.

## Data Availability

The data used to support the findings of this study are available from the corresponding author upon request.
